The article "Identification of Biomarkers for Predicting Allograft Rejection following Kidney Transplantation Based on the Weighted Gene Coexpression Network Analysis" was retracted in 2024. Reasons: signs of a paper mill; compromised peer review; unreliable results or conclusions.

# Identification of Biomarkers for Predicting Allograft Rejection following Kidney Transplantation Based on the Weighted Gene Coexpression Network Analysis

**DOI:** 10.1155/2021/9933136

**Published:** 2021-07-29

**Authors:** Li-Jun Wang, Xiao-Bo Ma, Hong-Ying Xia, Xun Sun, Lu Yu, Qian Yang, Zong-Qiang Hu, Yong-Heng Zhao, Wei Hu, Jiang-Hua Ran

**Affiliations:** ^1^Department of Urinary Surgery, The Affiliated Calmette Hospital of Kunming Medical University, The First People's Hospital of Kunming, Calmette Hospital, Kunming, Yunnan Province, China; ^2^Department of Clinical Laboratory, Yunnan Institute of Experimental Diagnosis, The First Affiliated Hospital of Kunming Medical University, Yunnan Key Laboratory of Laboratory Medicine, Kunming, Yunnan Province, China; ^3^Department of Pharmacy, Yan'an Hospital Affiliated to Kunming Medical University, Kunming, Yunnan Province, China; ^4^Department of Pathology, The Affiliated Calmette Hospital of Kunming Medical University, The First People's Hospital of Kunming, Calmette Hospital, Kunming, Yunnan Province, China; ^5^Department of Hepatopancreatobiliary Surgery, The Affiliated Calmette Hospital of Kunming Medical University, The First People's Hospital of Kunming, Calmette Hospital, Kunming, Yunnan Province, China

## Abstract

Kidney transplantation is the promising treatment of choice for chronic kidney disease and end-stage kidney disease and can effectively improve the quality of life and survival rates of patients. However, the allograft rejection following kidney transplantation has a negative impact on transplant success. Therefore, the present study is aimed at screening novel biomarkers for the diagnosis and treatment of allograft rejection following kidney transplantation for improving long-term transplant outcome. In the study, a total of 8 modules and 3065 genes were identified by WGCNA based on the GSE46474 and GSE15296 dataset from the Gene Expression Omnibus (GEO) database. Moreover, the results of Gene Ontology (GO) annotation and Kyoto Encyclopedia of Genes and Genomes (KEGG) pathway enrichment analysis showed that these genes were mainly involved in the immune-related biological processes and pathways. Thus, 317 immune-related genes were selected for further analysis. Finally, 5 genes (including CD200R1, VAV2, FASLG, SH2D1B, and RAP2B) were identified as the candidate biomarkers based on the ROC and difference analysis. Furthermore, we also found that in the 5 biomarkers an interaction might exist among each other in the protein and transcription level. Taken together, our study identified CD200R1, VAV2, FASLG, SH2D1B, and RAP2B as the candidate diagnostic biomarkers, which might contribute to the prevention and treatment of allograft rejection following kidney transplantation.

The article "Identification of Biomarkers for Predicting Allograft Rejection following Kidney Transplantation Based on the Weighted Gene Coexpression Network Analysis" was retracted in 2024. Reasons: signs of a paper mill; compromised peer review; unreliable results or conclusions.

## 1. Introduction

Kidney transplant is a promising method of kidney replacement therapy for chronic kidney disease and end-stage kidney disease [1, 2]. Increasing evidence has demonstrated that kidney transplantation can effectively improve the quality of life and survival rates of patients with chronic kidney disease and end-stage kidney disease [3]. However, the occurrence of allograft rejection following kidney transplantation greatly limits the success rate by resulting in degradation of kidney function and graft loss [4, 5]. Although the current advancements in the development of immunosuppressive medications targeting T cell-mediated immunity have effectively inhibited the occurrence of rejection reaction [6], the currently available immunosuppressive medications are ineffective against the adaptive humoral immune response. Moreover, to date, the detection of allograft rejection following kidney transplantation mainly relies on the biopsies, which is prone to misdiagnosis. Therefore, there is a continuing need for better understanding of the mechanism of allograft rejection following kidney transplantation and screening of novel biomarkers for the diagnosis and treatment of allograft rejection following kidney transplantation.

Currently, it has been suggested that understanding the underlying mechanisms of allograft rejection following kidney transplantation can contribute to identify potential therapeutic targets. Based on the key role of anti-HLA antibodies in the occurrence of rejection, many promising treatment methods have already being tested in clinical trials, such as B cell-depleting rituximab treatment and proteasome inhibition using bortezomib [7]. However, these treatment methods also have some limitations because of the individual heterogeneity [8]. Moreover, most therapies only focused on the immune cell level, a few studies on the molecular level [9, 10]. Recent researches have showed that CD20, VWF, and FOXP3 genes were upregulated in the peripheral blood of rejection patients [9]. Moreover, it has been raised that the expression of VWF, DARC, and CAV1 can effectively distinguish excluded rejection samples from nonrejection samples [10]. Therefore, genes especially immune-related genes may play a vital role in the occurrence of allograft rejection following kidney transplantation. Nevertheless, it remains largely unclear how these genes influence the occurrence of allograft rejection.

More and more approaches have been developed for identifying the disease-related modules and genes, which were highly effective for helping search for the diagnostic and therapeutic markers in clinical practice [11–14]. As an approach for screening disease-related modules, weighted gene coexpression network analysis (WGCNA) is the most common and useful method to reveal the association between genes and clinical features [15]. In previous study, WGCNA has been used to study the complex diseases, such as glioblastoma multiforme [16], cardiovascular disease in diabetic patients [17], and Sjögren's syndrome [18]. However, relative study in kidney transplant is still scarce.

The article "Identification of Biomarkers for Predicting Allograft Rejection following Kidney Transplantation Based on the Weighted Gene Coexpression Network Analysis" was retracted in 2024. Reasons: signs of a paper mill; compromised peer review; unreliable results or conclusions.

In the present study, kidney transplant gene expression data were downloaded from the NCBI Gene Expression Omnibus (GEO) database (https://www.ncbi.nlm.nih.gov/geo/query/acc.cgi). Next, WGCNA was constructed to identify rejection-related genes. Moreover, we further explored the potential molecular mechanism of rejection-related genes and provided the candidate biomarkers for the diagnosis of rejection, which will contribute to the therapy of allograft rejection following kidney transplantation.

## 2. Materials and Methods

### 2.1. Data Processing

Three kidney transplant-related gene datasets, including GSE46474, GSE15296, and GSE14067, were obtained from the NCBI GEO database. The detailed information of the three gene datasets is listed in Table 1. Next, GSE46474 and GSE15296 were combined as the training cohort, and GSE14067 was selected as the independent validation cohort. The batch effect between GSE46474 and GSE15296 was corrected with Limma [19] and SVA package [20] in R.

### 2.2. Construction of Gene Coexpression Network

WGCNA package [15] in R was selected to construct the weighted gene coexpression network based on all the genes involved in all samples in the training cohort. Firstly, we checked the association of all samples in the training cohort by performing sample cluster analysis and removed the outlier samples to ensure the accuracy of the analysis. Then, to ensure that the gene interaction maximally conforms to the scale-free distribution, we performed the soft threshold selection analysis to select the appropriate soft threshold. Moreover, hierarchical clustering was carried out to identify modules by a dynamic tree cutting algorithm with a minimum module size of 30 for the gene dendrogram [21]. Finally, the dissimilarity of module eigengenes (MES) was calculated for module dendrogram and some modules (the dissimilarity of module eigengenes < 0.25) were merged to obtain the ultimate network.

### 2.3. Identification of Rejection-Related Modules and Genes

To detect the independence between two different modules, we analyzed the association among different modules. Module eigengenes were used to evaluate the possible relationship between gene modules and clinical traits and to identify rejection-related modules. Finally, the genes in rejection-related modules were defined as rejection-related genes.

The article "Identification of Biomarkers for Predicting Allograft Rejection following Kidney Transplantation Based on the Weighted Gene Coexpression Network Analysis" was retracted in 2024. Reasons: signs of a paper mill; compromised peer review; unreliable results or conclusions.

### 2.4. Functional and Pathway Enrichment Analysis

Gene Ontology (GO) annotation, including biological processes (BP), molecular function (MF), and cellular component (CC), and Kyoto Encyclopedia of Genes and Genomes (KEGG) pathway enrichment analysis were performed to investigate the biological function of rejection-related genes by clusterProfiler package [22] in R, and *P* < 0.05 was considered to be significantly enriched. Besides, the results of enrichment analysis were plotted by ggplot2 package [23] in R.

### 2.5. Identification of Immune-Related Genes

Given the key role of immune immunoreaction in the allograft rejection following kidney transplantation, immune-related genes involved in the immune-related GO and pathways were selected and reserved for the subsequent analysis based on the results of enrichment analysis.

### 2.6. Differential Expression Analysis of Immune-Related Genes

The Wilcoxon rank sum test was used to identify differentially expressed and immune-related genes between rejection samples and nonrejection samples in the training cohort and the validation cohort, respectively, and *P* < 0.05 was considered to be statistically significant.

### 2.7. Identification of Hub Genes

Receiver operator characteristic curve was plotted using pROC package [24] in R to identify the hub genes based on the capability of distinguishing rejection samples and nonrejection samples in the training cohort which was evaluated by the area under the curve (ROC) value, and these genes with ROC > 0.7 were defined as hub genes.

### 2.8. PPI Network Construction and Gene Correlation Analysis

To further investigate the interactions between hub genes and other rejection-related genes at the protein level, the Search Tool for the Retrieval of Interacting Genes (STRING, https://string-db.org/) was used to build the protein-protein interaction (PPI) network. Next, Cytoscape version 3.7.1 [25] was used to visualize and analyze the interactions of the proteins, and the cutoff value was set to confidence = 0.4. Moreover, psych package in R was used to compare the association between any two hub genes.

### 2.9. Statistical Analysis

Statistical analysis was performed using R software v 4.0.2. Unless otherwise stipulated, *P* < 0.05 was considered statistically significant.

## 3. Results

### 3.1. Identification of Gene Coexpression Networks

The results of batch correction clearly showed that the batch effect between GSE46474 and GSE15296 was effectively eliminated and the combined dataset, including 44 nonrejection samples and 71 rejection samples, could be used for further analysis (Figure 1). Next, the sample cluster analysis showed that GSM382283 was an outlier sample in the combined dataset. Hence, GSM382283 was removed and remaining samples were used for subsequent analysis (Figure 2(a)). To construct a scale-free network, soft threshold selection analysis suggested that *β* = 7 (scale free *R*^2^ = 0.90) was optimal soft thresholds (Figure 2(b)). Finally, by setting the dissimilarity of module eigengenes < 0.25, 24 modules were identified (Figure 2(c)).

The article "Identification of Biomarkers for Predicting Allograft Rejection following Kidney Transplantation Based on the Weighted Gene Coexpression Network Analysis" was retracted in 2024. Reasons: signs of a paper mill; compromised peer review; unreliable results or conclusions.

### 3.2. Association between Any Two Modules and Identification of Hub Modules

To further quantify the coexpression similarity among 27 modules, the correlation between any two modules was calculated, and the results suggested that 27 modules could be divided into two main clusters based on their correlation (Figure 3(a)). Moreover, we also randomly selected 400 genes to construct the gene cluster tree and to plot the network heat map. Based on the heat map plot, we could see that each module showed independence to other modules. Therefore, the 27 modules were effective and representative (Figure 3(b)). In our study, nonrejection and rejection were selected as two clinical parameters to identify rejection-related modules. Based on *P* < 0.05, blue module, cyan module, dark turquoise module, grey60 module, ivory module, pale turquoise module, saddle brown module, and yellow green module were selected as the rejection-related modules and 3065 genes in these 8 modules were defined as rejection-related genes (Figure 3(c)).

### 3.3. Functional and Pathway Enrichment Analysis

To further investigate the GO function and KEGG pathways which involved rejection-related genes, functional and pathway enrichment analysis was performed using the clusterProfiler package in R. The GO enrichment results showed that for BP, the rejection-related genes were mainly associated with T cell activation, T cell differentiation, and positive regulation of defense response; for CC, the rejection-related genes were mainly related to tertiary granule; and that for MF, the rejection-related genes were mainly involved in activation of immune receptors and chemokine receptor binding (Figure 4(a), Supplementary material 1). In addition, the results of KEGG pathway enrichment analysis also showed that rejection-related genes were mainly related to the interaction of viral proteins with cytokines and cytokine receptors, osteoclast differentiation, and immune-related pathways, for example, natural killer cell-mediated cell toxicity, IL-17 signaling pathway, and T cell receptor signaling pathway (Figure 4(b), Supplementary material 2). Hence, these results indicated that these genes might mediate the rejection by activating immune-related pathways.

The article "Identification of Biomarkers for Predicting Allograft Rejection following Kidney Transplantation Based on the Weighted Gene Coexpression Network Analysis" was retracted in 2024. Reasons: signs of a paper mill; compromised peer review; unreliable results or conclusions.

### 3.4. Identification of Differentially Expressed and Immune-Related Genes

Based on the results of functional and pathway enrichment analysis, 317 immune-related genes which were involved in immune- and inflammation-related GO function and immune-related pathways were extracted for further analysis. The results of the Wilcoxon rank sum test showed that 96 immune-related genes were significantly differentially expressed in rejection samples compared to nonrejection samples in the training cohort. Moreover, 121 immune-related genes were significantly differentially expressed in rejection samples compared to nonrejection samples in the validation cohort. Thus, after overlapping the differentially expressed and immune-related genes in the training cohort and the validation cohort, 45 differentially expressed and immune-related genes were selected for subsequent analysis (Figure 5).

### 3.5. Identification of Hub Genes

To further identify the hub genes which could effectively distinguish rejection samples and nonrejection samples, ROC curves of 45 genes were plotted to evaluate the capacity of genes in rejection samples and nonrejection samples. Finally, based on the AUC value of each gene, 6 genes including CD200R1, MIR142, VAV2, FASLG, SH2D1B, and RAP2B were identified as hub genes because they could better distinguish rejection samples and nonrejection samples (AUC > 0.7, Figure 6). Notably, only 5 genes (including CD200R1, VAV2, FASLG, SH2D1B, and RAP2B) showed the consistent expression trends between the training cohort and the validation cohort (Figures 7(a), 7(c), and 7(d)–7(f)), but MIR142 showed the opposite expression trends between the training cohort and the validation cohort (Figure 7(b)). Thus, CD200R1, VAV2, FASLG, SH2D1B, and RAP2B were retained as the candidate diagnostic biomarkers.

### 3.6. PPI Network Construction and Gene Correlation Analysis for Hub Genes

To further investigate the interactions between candidate diagnostic biomarkers and other rejection-related genes in protein levels, the PPI network was constructed for all immune-related genes using the STRING database. The result of PPI network showed that all 5 candidate diagnostic biomarkers had existing interactions with other proteins (Figure 8(a)). Thus, the alterations in protein levels for the 5 genes might influence the expression level of other proteins resulting in the occurrence of rejection. Moreover, we also calculated the association of the expression for candidate diagnostic biomarkers in the training cohort. Surprisingly, we found that SH2D1B had a strong positive correlation with FASLG and RAP2B, which could suggest that the expression of them might influence each other (Figure 8(b)).

The article "Identification of Biomarkers for Predicting Allograft Rejection following Kidney Transplantation Based on the Weighted Gene Coexpression Network Analysis" was retracted in 2024. Reasons: signs of a paper mill; compromised peer review; unreliable results or conclusions.

## 4. Discussion

Currently, allograft rejection following kidney transplantation has been regarded as a main cause of graft failure after kidney transplantation [26–28], and the diagnosis of allograft rejection following kidney transplantation primarily relied on the histological examination of a kidney biopsy [29]. However, kidney biopsy also had many errors. Moreover, although other diagnosis biomarkers for allograft rejection have also been researched, few biomarkers were identified in clinical practice. Therefore, novel biomarkers in the molecular level are essential for improving the early diagnosis and therapy of allograft rejection.

In the present study, 3065 rejection-related genes were identified based on WGCNA. The result of GO and KEGG enrichment analysis showed that these genes were mainly involved in the immune-related biological processes and pathways. Thus, 317 immune-related genes were preserved for further analysis. Finally, based on the difference analysis and ROC analysis, 5 genes (including CD200R1, VAV2, FASLG, SH2D1B, and RAP2B) were selected as the candidate diagnostic biomarkers (Figures 6 and 7).

It has been demonstrated that allograft rejection was related to molecular changes [30, 31]. Our study found that the expression of CD200R1, VAV2, FASLG, SH2D1B, and RAP2B was both dissonant in rejection samples compared with nonrejection samples between the training cohort and the validation cohort, which further elucidated that the occurrence of allograft rejection following kidney transplantation was associated with the molecular changes. Consistent with our results, CD200R1, a member of the immunoglobulin superfamily, has been proved to predict immunosuppression and high-risk severity after kidney transplantation [32]. Therefore, CD200R1 might play a key role in allograft rejection. VAV2 was confirmed to affect alloreactivity and allograft survival in mice [33]. Our study suggested for the first time that VAV2 was associated with allograft rejection following kidney transplantation in humans. FASLG was found to be upregulated in renal transplant recipients after the treatment of cyclosporine (CsA) and tacrolimus (FK506) [34]. Hence, FASLG was promising to become a therapeutic target for allograft rejection following kidney transplantation. In addition, SH2D1B has already been proposed to be associated with the antibody-mediated rejection in kidney transplantation and could be selected as a predictor for graft loss [35]. As for the rest of the hub genes, RAP2B was not reported to be related to allograft rejection following kidney transplantation. Moreover, we also explored the relationships of protein interactions between 5 candidate diagnostic biomarkers and other immune-related genes and found that 5 candidate diagnostic biomarkers have interactions with other proteins (Figure 8(a)). Furthermore, we also found that there were strong correlations among FASLG, SH2D1B, and RAP2B in the transcriptional level (Figure 8(b)). Hence, we speculated that these genes might influence each other in the transcriptional level resulting in the occurrence of allograft rejection.

The article "Identification of Biomarkers for Predicting Allograft Rejection following Kidney Transplantation Based on the Weighted Gene Coexpression Network Analysis" was retracted in 2024. Reasons: signs of a paper mill; compromised peer review; unreliable results or conclusions.

As expected, these genes are mainly related to immune-related biological processes and pathways (Figure 4, Supplementary materials 1 and 2). Immune response has been considered as a major cause of graft loss [36, 37], resulting in the patients' need to receive immunosuppressive drug regimens [37]. Although all kinds of immune cells can contribute to graft rejection and failure, T cell- and antibody-mediated rejection usually in acute and chronic rejection has the major role [27]. Our study found that 5 candidate diagnostic biomarkers were mainly related to T cell activation and differentiation. Hence, we speculated that theses 6 genes might affect allograft rejection by activating T cell-related pathways.

## 5. Conclusion

In summary, the present study identified 6 immune-related genes that were associated with allograft rejection following kidney transplantation. Although additional researches are needed to demonstrate the roles for these gens, it is promising that the findings will contribute to understand the molecular mechanism of allograft rejection following kidney transplantation. Therefore, our study will conduce to the prevention and treatment of allograft rejection following kidney transplantation.

## Figures and Tables

**Figure 1:** The batch effect correction of GSE46474 and GSE15296. (a) The distribution of gene expression for the samples before correction. (b) The distribution of gene expression for the samples after correction.

**Figure 2:** Gene coexpression network construction. (a) Sample cluster analysis identified GSM382283 as the outlier samples in the training cohort. (b) Soft threshold selection analysis to select the appropriate soft threshold. (c) 24 modules were identified by setting the dissimilarity of module eigengenes < 0.25.

**Figure 3:** Module correlation analysis. (a) Module clustering and heat map of the eigengene adjacency. (b) Gene clustering results by random selection of 400 genes. (c) Module correlation analysis.

**Figure 4:** GO functional annotation and KEGG pathway enrichment analysis for the rejection-related genes. (a) Bar diagram shows the top 10 GO terms enriched by the rejection-related genes. (b) Bubble plots show the top 10 KEGG pathways enriched by the rejection-related genes.

The article "Identification of Biomarkers for Predicting Allograft Rejection following Kidney Transplantation Based on the Weighted Gene Coexpression Network Analysis" was retracted in 2024. Reasons: signs of a paper mill; compromised peer review; unreliable results or conclusions.

**Figure 5:** Overlapping and differentially expressed immune-related genes in the training cohort and the validation cohort identified by the Wilcoxon rank sum test.

**Figure 6:** ROC analysis identification of hub genes in the training cohort: (a) CD200R1, (b) MIR142, (c) VAV2, (d) FASLG, (e) SH2D1B, and (f) RAP2B.

**Figure 7:** The gene expression of hub genes in the training cohort and the validation cohort: (a) CD200R1, (b) MIR142, (c) VAV2, (d) FASLG, (e) SH2D1B, and (f) RAP2B.

**Figure 8:** The PPI network and association of 5 candidate diagnostic biomarkers. (a) PPI network for the 5 candidate diagnostic biomarkers. (b) The association of 5 candidate diagnostic biomarkers.

**Table 1:** The information of three transplant-related gene datasets from the GEO database.

GEO number	Rejection	Nonrejection	Platforms	Description
GSE46474	20	20	GPL570	Affymetrix Human Genome U133 Plus 2.0 Array
GSE15296	51	24	GPL570	Affymetrix Human Genome U133 Plus 2.0 Array
GSE14067	38	37	GPL570	Affymetrix Human Genome U133 Plus 2.0 Array

## Data Availability

All data are available in this paper.

## Supplementary Materials

Supplementary Materials Supplementary material 1: all GO terms enriched by the rejection-related genes. Supplementary material 2: all KEGG pathways enriched by the rejection-related genes.
